# Depot-specific differences in fat mass expansion in WT and *ob/ob* mice

**DOI:** 10.18632/oncotarget.17938

**Published:** 2017-05-16

**Authors:** Xinxia Wang, Caihua Yu, Jie Feng, Jin Chen, Qin Jiang, Shihuan Kuang, Yizhen Wang

**Affiliations:** ^1^ College of Animal Sciences, Zhejiang University, Key Laboratory of Animal Nutrition & Feed Sciences, Ministry of Agriculture, Zhejiang Provincial Laboratory of Feed and Animal Nutrition, Hangzhou, Zhejiang 310058, P. R. China; ^2^ Department of Animal Sciences and Center for Cancer Research, Purdue University, West Lafayette, IN 47907, USA

**Keywords:** adipogenesis, subcutaneous adipose tissue, viseral adipose tissue, fatty acid uptake, β-oxidation

## Abstract

The study was designed to investigate the cellular mechanisms underlying the differential fat expansion in different fat depots in wild type (WT) and *ob/ob* (OB) mice. At 6 weeks old, no differences in fat mass were found between SAT and VAT in WT mice, while O-SAT showed significantly higher weight than that of O-VAT. The average adipocyte size of SAT (∼ 4133.47 μm^2^) was smaller than that of VAT (∼ 7438.91 μm^2^) in OB mice. O-SAT preadipocytes gained higher triglyceride contents and higher levels of PPARγ and C/EBPα than did O-VAT preadipocytes upon *in vitro* differentiation. W-SAT and W-VAT displayed no significant differences in fatty acid uptake, while 1.36 fold significantly higher fatty acid uptake was found in O-SAT compared to O-VAT. Approximately 52% of the radioactivity recovered in cellular lipids was found in TAG in O-SAT, which was significantly higher than the other three adipocyte types. Significantly more radiolabelled oleic acid was β-oxidized to CO2 in adipocytes from O-VAT than that from O-SAT. ATP production was significantly lower in W-SAT compared with W-VAT, whereas no significantly ATP level was observed between O-SAT and O-VAT. Expression of UCP-1 in SAT from either WT or OB mice was significantly higher than the counterpart of VAT, which demonstrated higher uncoupled respiration and lower oxidative phosphorylation in SAT. Together, a combined increase in adipogenesis and FA uptake, and decreases in β-oxidation and ATP production, contributed to greater expansion of SAT compared to VAT in obese mice.

## INTRODUCTION

Over the past decades years, the prevalence of obesity has increased dramatically and scientists have realized that not all adipose tissue is alike [1]. The health risk is associated with the location as well as the amount of body fat. Adipose tissue, appear in multiple locations throughout the body, serves as an important regulator of metabolic homeostasis. Regional differences in the fat mass accumulation, both in visceral and subcutaneous areas, lead to remarkable differences in body fat distribution. The distribution of fat has clinical importance, as central adiposity, especially visceral obesity, is associated with insulin resistance and a high risk for type 2 diabetes and metabolic syndrome, whereas accumulation of subcutaneous fat has been shown to have a possible protective value against these metabolic abnormalities [2].

During weight gain, accumulation of regional adipose tissue is determined by hyperplasia, hypertrophy, or a combination of both [3]. New adipocytes can be generated more rapidly in some depots than others [4]. A majority of studies reported that subcutaneous preadipocytes had a greater adipogenic capacity than did visceral cells. Blouin et al. reported subcutaneous (SC) preadipocytes had higher differentiation rates compared with omental (OM) adipose tissuecells [5]. Tchkonia et al. reported subcutaneous preadipocytes, which had the highest lipid accumulation, G3PD activity and aP2, PPARγ and C/EBPα expression than omental adipose tissue. The proportion of differentiated cells in colonies derived from single subcutaneous preadipocytes was higher than in omental clones [6]. It was studied that omental preadipocytes responded less well to the prodifferentiating effects of thiazolidinediones than do preadipocytes from subcutaneous (SC) depots [7]. Preadipocytes of the subcutaneous fat depot appear to be more responsive to adipogenic stimulation compared with those from visceral fat compartments in most studies [8]. A higher adipogenic capacity of subcutaneous preadipocytes than omental preadiocytes originating from the same women was observed [9]. Cultured human abdominal subcutaneous preadipocytes accumulate lipid, express markers of adipogenesis and adipogenic transcription factors to a greater extent than omental cells [10, 11]. However, no significant differences were also observed between SC and OM preadipocytes differentiation [12, 13]. Regional differences in preadipocyte replication, differentiation, subtype abundance, susceptibility to apoptosis or senescence, and gene expression may contribute to regional variation in fat-tissue function [4], a speculation that requires more research to test. Although the differences in terms of the gene expression signatures in SAT and visceral adipose tissue (VAT) have been described [8, 14], the cellular mechanism underlying the difference in fat mass accumulation is unclear.

The aim of this study was to investigate cellular mechanisms underlying the differential expansion of SAT and VAT inmice. To this end, we determined the size of mature adipocytes, variations in differentiation capacity, FA uptake, mitochondria functions in SAT and VAT depots in lean and obesemice. Understanding the mechanism of regional fat mass expansion may facilitate developing strategies for modulating fat distribution and influencing whole-body metabolism.

## RESULTS

### Differences in SAT and VAT expansion in obese and lean mice

To confirm the obesogenic effect of the *ob/ob* mouse model used in this study, we first compared the body weight of WT and *ob/ob* mice. At 6 weeks old, the *ob/ob* mice weighted 2.5 times as heavy as the WT mice (40.52 ± 0.43g vs16.11± 0.23 g, respectively, *P*< 0.05) (Figure 1A). To further determine the differences in fat mass of various depots, we analyzed the inguinal fat (a depot ofSAT) and epididymal fat (a depot of VAT). In WT mice, no significant differences in fat mass were found between SAT and VAT, while SAT showed significantly higher weight than that of VAT in *ob/ob* mice (Figure 1B). On average, the SAT and VAT mass expanded by 29.4 and 12.7 fold, respectively in the *ob/ob* mice compared to WT mice. To determine whether SAT and VAT expansion via different mechanisms in obese mice, we measured adipocytes size in both depots harvested from WT and*ob/ob* after hematoxylin and eosin (H&E) staining. Obese mice had an average 5.82 fold increase (from 710.52±12.22 μm^2^ to 4133.47±153.11 μm^2^, n > 200) in adipocytes area in SAT compared with 7.92 fold increase (from 945.06±20.96 μm^2^ to 7438.91±153.10μm^2^, n > 200) in VAT (Figure 1C, 1D), suggesting that VAT expanded by adipocytes hypertrophy, which was in agreement with other studies [15]. Since we found SAT gained higher fat mass (Figure 1B) than VAT, adipocytes hyperplasia must play a greater role in SAT than in VAT expansion. Adipogenesiswas the process resulting in adipose tissue hyperplasia [16], therefore, we next tested the adipogenesis capacity in SAT and VAT.

**Figure 1:** Differences in SAT and VAT expansion in obese and lean mice Body weight of WT and *ob/ob* mice at 6 weeks of age **(A)**, Fat mass in both depots from WT and ob/ob mice **(B)**, H&E staining of adipocyte **(C)** and Adipocyte size (n > 400 adipocytes) **(D)**. Data are shown as means ± s.e.m (n=4), * *P*< 0.05, ** *P*< 0.01.

### O-SAT showed higher adipogenesis capacity than O-VAT

White adipose tissue was a complex material which contains different cell types. So SVFs represents a physiologically more relevant model for preadipocyte differentiation than pure adipocyte precursor cells (APCs). To evaluate adipogenesis capacity of the preadipocytes in culture, both TAG contents assay and ORO staining were conducted. After exposure to differentiation medium for 6 days, cells exhibited no significant difference in lipid accumulation between two adipose depots from lean mice (W-SAT and W-VAT), while O-SAT (SAT from *ob/ob* mice) accumulate more lipid than O-VAT (VAT from *ob/ob* mice) (Figure 2A). ORO staining and OD value from ORO staining showed the similar results (Figure 2B, 2C). Terminal differentiation of preadipocytes into mature, lipid-storing cells were a complex process principally controlled by two major transcription factors, PPARγ and C/EBPα [16]. PPARγ and C/EBPα showed no significant differences between W-SAT and W-VAT, while exhibited significantly higher expression in O-SAT compared to O-VAT (Figure 2D, 2E), suggesting O-SAT had a higher capacity to accumulate lipid than O-VAT. These results supportedthat greater adipogenesis capacity was found in SAT than VAT in obese mice.

**Figure 2:** Adipogenesis capacity of preadipocytes Preadipocytes from mice were induced into mature adipocytes and harvested on day 6. TAG content in adipocytes from W-SAT, W-VAT, O-SAT and O-VAT **(A)**, Oil red O (ORO) staining of adipocytes (200×) **(B)**, OD value quantification of ORO staining **(C)**, PPARγ and C/EBPα mRNA expression **(D, E)**. Data are shown as means ± s.e.m (n=4), * *P*< 0.05, ** *P* < 0.01.

### O-SAT uptook more fatty acids, but showed lower β-oxidation than O-VAT

To explore the cellular mechanisms of adipogenesis capacity, the respectivecapacities for FAs uptake were evaluated in adipocytes from different fat depots incubated with [1-^14^C]OA. Results showed the total disintegrations per minute (dpm) of [1-^14^C]OA recovered in cellular lipids in adipocytes (Figure 3). No significant differences in fatty acid uptake were observed in W-SAT and W-VAT, while 1.36 fold significantly higher in fatty acid uptake was found in O-SAT compared to O-VAT (Figure 3A). Genes expression showed that FABP4, ACBP and ACSL-1 were significantly higher in O-SAT than the other three adipocyte types, which was in agreement with results of fatty acid uptake (Figure 3D, 3E, 3F). One of fate of the fatty acidsthat adipocytesuptook were locally re-esterified in cells. To examine the differences infatty acid re-esterification into various lipid classes, the relative incorporations of radiolabelled [1-^14^C]OA in the different intracellular lipid classes, such as phospholipid (PL), free fatty acid (FFA), triacylglycerols (TAG), Diacylglycerols (DAG) and cholesteryl ester (CE) were analyzed byHPTLC. For W-SAT, W-VAT and O-VAT, more than 50% of the radioactivitieswere found in PL, while about30% was recovered in TAG. Approximately 52% of the radioactivity recovered in cellular lipids was found in TAG in the O-SAT, which was significantly higher than the other three adipocyte types (*P*< 0.05, Figure 3B).

**Figure 3:** FAs uptake, β-oxidation and relative distribution of radioactivity from [1-^14^C] OA in cellular lipids Adipocytes were incubated with radiolabeled OA for 24h. Cellular fatty acid uptake **(A)**, Relative distribution of [1-^14^C] OA in lipid classes **(B)**, β-oxidation **(C)** and mRNA Expression of FABP4, ACBP, ACSL-1, FATP1, COX IV **(D, E, F, G, H)**. Data are shown as means ± s.e.m (n=4), * *P*< 0.05, ** *P*< 0.01.

In addition to re-esterification, some of the fatty acidswere oxidized in cells after they were taken in. To show the differences in fatty acid β-oxidation between fat-depots, ^14^CO_2_were collected after the treatment of cells with [1-^14^C]OA. The results showed that fat-depots from obese mice exhibited significantly lower β-oxidation rate than those from WT mice (*P*< 0.05). For regional adipose tissue, no significant differences were observed between W-SAT and W-VAT, while significantly more radiolabelled OA was β-oxidized to CO_2_ in adipocytes from O-VAT (6951.6±434.6 dpm/mg protein, 0.21% of total uptake) than that from O-SAT (3328.7±145.7 dpm/mg protein, 0.07% of total uptake) (*P*< 0.01, Figure 3C). Genes related to fatty acid β-oxidation were quantified. Significantly lower FATP1 and COX IV expression were observed in *ob/ob* than those in WT mice (*P*< 0.05). There was no significant difference in FATP1 expression between SAT and VAT either from *ob/ob* or WT mice (*P*> 0.05). W-VAT showed significantly higher COX IV expression compared with W-SAT (*P*< 0.05), although no difference was observed between O-SAT and O-VAT (*P*> 0.05, Figure 3G, 3H).

### The lowerFFA β-oxidation in O-SAT wasunlikely related to mitochondrial function

Since fatty acid β-oxidation occurred in mitochondrial matrix, mitochondrial function in various fat-depots was examined. The predominant physiological function of mitochondria was the generation of ATP by oxidative phosphorylation, and mitochondrial function is often assessed by the ability to produce ATP appropriately [17]. Our results showed adipose tissue from obese mice produced significantly less ATP than those from WT mice. For regional fat-depots, ATP production was significantly lower in W-SAT compared with W-VAT (*P*< 0.05). No significantly ATP level was observed between O-SAT and O-VAT (Figure 4A). ATP was generated by oxidative phosphorylation (OXPHOS) through electron transport chain, which is composed by enzymes of complex I, II, III, IV and V. The expressions of these enzymes are also markers representing mitochondrial function. In this study, relatively lower expressions of complex I, II, III, IV and V were found in adipose tissue from *ob/ob* mice compared to WT mice (Figure 4C). No significant difference was observed of complex I and IV between W-SAT and W-VAT, whereas the expression of complex Iand IV showed significantly decreased in O-VAT than O-SAT (Figure 4C, 5A, 5C). To further explain the paradox of the ATP production and OXPHOS between regional fat-depots, uncoupling protein 1 (UCP-1) was detected. Expression of UCP-1in SAT from either WT mice or *ob/ob* micewas significantly higher than the counterpart of VAT (Figure 4B), which demonstrated higher uncoupled respiration and lower oxidative phosphorylation in SAT.

**Figure 4:** Mitochondrial function in different depots from WT and *ob/ob* mice Cellular ATP content **(A)**, Expression of UCP-1 **(B)** and Enzymes of oxidative phosphorylation (OXPHOS) complex I, II, III, IV and V **(C)**. β-actin was used as a loading control (n=5). Data are shown as means ± s.e.m (n=4), * *P*< 0.05, ** *P*< 0.01.

**Figure 5:** Relative protein expression of oxidative phosphorylation (OXPHOS) complex I, II, III, IV and V **(A, B, C, D, E)**. Data are shown as means ± s.e.m (n=3), * P< 0.05, ** P< 0.01.

## DISCUSSION

In this study, we compared the differences in body weight gain and body fat distribution in the setting of obesity in obese mice. The results showed obese mice had significantly higher body weight and this weight gain mostly resulted from an increase in fat tissue. Fat mass in different location increased differently. SAT gained much more weight than VAT during obesity. To explore the mechanisms responsible for regional variation in fat mass expansion, we investigated the differences in regional adipocyte size. Adipocytes in VAT grew larger than those in SAT in obese mice, which in line with the results from mice with HFD-induced obesity [18]. The significantly larger VAT adipocyte size suggested that VAT expanded by adipocyte hypertrophy, which was in agreement with other studies [15]. In our study, the higher fat mass gained and smaller adipocytes in SAT than VAT with onset of obesity indicated adipocytes hyperplasia play a greater role in SAT than in VAT expansion in obese mice. It had been reported that in rat, the capacity of preadipocyte proliferation and recruitment was higher in SAT than VAT depots [19]. Adipogenesis was the process resulting in adipose tissue hyperplasia [16], we next compared the adipogenesis capacity in SAT and VAT from WT and *ob/ob* mice.

Studies from human showed that adipogenesis capacity varied among fat depots [6, 16]. Human abdominal SAT preadipocytes had a greater capacity for adipogenesis than omental cells [6, 16]. In mice study, higher differentiation capacity was observed in adipocyte precursor cells (APCs) from SAT than from VAT depots [8]. In our study, no significant difference was observed in adipogenesis capacity in fat-depots from WT mice. However, O-SAT showed significantly higher adipogenesis capacity than O-VAT, which may partly explain the greater fat mass gained in SAT than those in VAT in obese mice. Adipogenesis were involved in the sequential induction of multiple transcription factors. In our study, mRNA levels of PPARγ and C/EBPα increased significantly in O-SAT compared with O-VAT, in line with previous reports [6, 20]. Our current findings suggested the different responses of SAT or VAT in adipogenesis led to their different contributions to obesity or metabolic disorders. Higher adipogenesis in SAT seemed to be beneficial from the metabolic standpoint as it predicted a better metabolic profile, most likely due to increased lipid storage capacity. It remained to be clarified whether the lower ability for VAT to differentiate compared with their SAT counterparts reflected the depot's effects on the development of metabolic disorders.

Regional differences in free fatty acid (FFA) handling including fatty acid uptake, re-esterification or FFA releases between various fat depots contributed to body fat distributions [21]. Studies showed differences in FFA releases (lipolysis) did not explain variations in body fat distribution [22, 23]. Regional differences in fatty acid uptake could potentially account for the differences in body fat distribution [24]. *In vivo* studies of meal FA uptake provided definitive evidence for heterogeneity in the metabolism of VAT and SAT. Expressed relative to the same mass AT, meal FA uptake was greater in intra-abdominal than abdominal SAT in both sexes [24]. The direct uptake of plasma FFA was also greater (per unit mass) in omental compared to abdominal SC of women [25]. However, on a per cell basis, uptake and esterification may be similar or even lower in visceral adipocytes because there were more adipocytes per gram. Studies from Jesen's group proposed that direct FFA uptake rather than meal fat uptake or lipoytic rates may explain sex-dependent body fat distribution [25]. Fatty acid uptake and storage had been well studied *in vivo*, but limited information was available in adipocytes. In our studies, no significant difference was observed in direct FFA uptake expressed by per milligram protein between W-SAT and W-VAT, while O-SAT took up significantly higher FFA compared with O-VAT. It had been reported that FFA uptake and storage per million low-body subcutaneous (LBSQ) adipocytes were positively associated with LBSQ fat mass [26], and LBSQ adipocytes stored more FFA in women with greater adiposity [26]. Therefore, the higher FA uptake in O-SAT may contribute to higher fat mass in SAT from *ob/ob* mice. Higher upregulation of FABP4 (aP2), ACBP and ACSL-1 confirmed the results from fatty acid uptake experiment *in vitro*. O-SAT exhibited significantly higher proportion of fatty acid uptook re-esterifed into TAG compared with W-SAT, W-VAT and O-VAT, further confirming another suggested role of SAT to be a buffer during intake of dietary lipids, thus protecting other tissues from lipotoxic effects [44].

Our study also showed fatty acid β-oxidation was decreased in the setting of obesity, which in agreement with previous studies in *ob/ob* mice that showed a reduction in the metabolic rate and a marked decrease in energy expenditure [27, 28]. Another study in our group also proved the less oxidation in obese mice than in lean mice by using radiolabelled fatty acid [29]. With regard to regional differences, no significant difference was observed between SAT and VAT in WT mice, while O-SAT showed significantly lower β-oxidation than O-VAT. VAT was bioenergetically more active than SAT in rat [30]. In obese human, visceral fat has been shown to be more metabolically active than subcutaneous fat [31, 32]. SAT was less metabolically active than VAT, it may have better short-term and long-term storage capacity [33]. Thus, this depot was important to accumulate TAG in periods of excess energy intake and supply the organism with FFAs in periods of fasting, starvation, or exercise.

Studies showed differences in metabolic activity may due to different mitochondrial function [30]. The significantly lower ATP content and apparent lower complex I-V expression in obese mice compared with lean mice suggesting mitochondria dysfunction in obese mice. Large studies tied the suboptimal function of mitochondria to obesity and T2DM. In patients with insulin resistance, T2DM, and severe obesity, the abundance of mitochondria and the expression of key genes pertinent to mitochondrial function are significantly decreased in WAT [34], in concert with reduced adipocyte oxygen consumption rates and ATP production [35]. The levels of approximately 50% of gene transcripts encoding mitochondrial proteins were decreased with the onset of obesity [36]. Furthermore, microarray profiling studies have revealed that genes crucial for mitochondrial function and OXPHOS were downregulated in obese, high-fat diet (HFD)-fed, insulin-resistant mice, and in *db/db* mice [37, 38]. With regard to regional differences, significantly higher ATP production in W-VAT was observed compared to W-SAT, which in agreement with studies in human that OXPHOS activity was significantly higher in VAT compared with SAT. Adipocytes from rat epididymal also showed higher respiratory rates than inguinal adipose tissue [30]. Although no significant difference in ATP content was found between O-SAT and O-VAT, OXPHOS enzymes, especially complex I and IV, reduced in O-VAT compared with O-SAT. This was confirmed by studies in which expression of genes belonging to the ETC has been shown to be decreased in VATcompared with SAT in obesity and insulin-resistant humans [39]. To further explain the paradox of the ATP production and OXPHOS between regional fat-depots, uncoupling protein 1 (UCP-1), which mediated heat generation and low rate of ATP production, was detected. Results showed higher expression was observed in SAT from either WT mice or *ob/ob* mice, which can partly explain the relative low ATP production in W-SAT, and no higher in ATP production in O-SAT with higher expression of OXPHOS enzymes.

In conclusion, the much greater mass of SAT compared to VAT may certainly result from higher adipogenesis, free FAs uptake, lower β-oxidation and ATP production, which in turn resulted in generation of new fat cells and additional lipid accumulation in SAT. These findings suggested that, in the setting of obesity, an enhanced capacity of fat mass expansion in SAT may prevent VAT enlargement and systemic lipotoxicity, which could be protective for metabolic syndromes. Together with differences in capacities for fat mass expansion, there were intrinsic interdepot differences in preadipocytes functional characteristics. Additional studies were needed to elucidate how extrinsic and environmental factors interacted with the innate properties of adipocytes under normal conditions and in disease states.

## MATERIALS AND METHODS

### Ethics statement

All procedures were approved by the Committee on Animal Care and Use and Committee on the Ethics of Animal Experiments of Zhejiang University. The protocol number was ZJU2015-458-09.

### Animals

Female lean wild type (WT) C57BL/6J and obese C57BL/6J *ob/ob* mice from same parents at 6 wk of age were purchased from Nanjing Biomedical Research institute of Nanjing University and maintained in barrier facility (12:12h light-dark cycle) with *ad libitum* access to food and water. The diet consisted of 10% (kcal%) fat from lard and soybean oil, 20% protein and 70% carbohydrate.

### Histology sampling

Subcutaneous and perigonadal fat pads, representing SAT and VAT, from three lean and obese mice (6wk) were takenat the same time, fixed in 4% buffered formalin, dehydrated in a graded ethanol series and embedded in paraffin. Sections (4μm) were stained with haematoxylin and eosin and observed under light microscopy (1).

### Cell isolation and differentiation

Subcutaneous and perigonadal fat pads, representing SAT and VAT, respectively, were isolated from lean and obese mice (6wk) and minced into small pieces and digested using 1 mg/ml collagenase I (Gibco, MD, USA) for isolation of preadipocytes. After removing large particles, the resulting suspension was centrifuged and the sediment cells resuspended in a growth medium (GM) were seeded in plates. Two days after postconfluence (d 0), the cells were stimulated to differentiate with differentiation medium (DM) (DM: GM, 0.5μmol/l 3-isobuty-1-methylxanthine (IBMX), 1μmol/l dexamethasone, and 167 nmol/l insulin) for 2 d (d 2), then maintained in 10% FBS/DMEM medium with 167 nmol/L insulin for another 2 d (d 4), followed by culturing with GM until analysis. To visualize the accumulated triacylglycerol in the adipocytes after differentiation, the cells were stained with ORO according to Wang et al. (2).

### Measurement of ^14^CO2 from [1-^14^C] FAs β-oxidation

Adipocytes (day 6) were incubated with 10μM (1.65 μci) of [1-^14^C] 18:1n-9 (American Radiolabeled Chemicals, Saint Louis, MO, USA) at 37°Cfor 24h. The medium from each cell well was used to analyze the amount of ^14^CO_2_ produced as described by Christiansen et al. (27). The 1.5 ml medium were transferred to a sealed glass vial with a center well containing a Whatman filter (pore size, Æ 125mm) paper moistened by adding 0.3 ml of phenylethylamine/methanol (1:1, v/v) (freshly made) with a 1 ml syringe end. The medium was acidified with 0.3ml 1M perchloric acid by injecting the acid with a syringe to cell medium. After incubation for 1h at room temperature, the wells containing the filter papers were placed into vials and dissolved with 5 ml of liquid scintillation fluid for scintillation counting. The cells were harvested and stored at -40°C prior to the extraction of lipid and analysis of radiolabeled lipid classes.

### Measurement of ASP from [1-^14^C] FAs

The 0.4mL medium was acidified with 0.2mLperchloric acid (2M) and then incubated for 60 min at 4°C. The medium was then centrifuged and the supernatant was used for scintillation counting.

### Measurement of [1-^14^C] FAs uptake

Adipocytes were washed by PBS for six times and PBS was removed completely. Cells were harvested with 1mL methanol and sonicated for 30 sec to get 1ml “methanol-cell solution”. 50μL methanol-cell solution was taken anddissolved with 5 ml of liquid scintillation fluid for scintillation counting. 0.2mL methanol-cell solution was taken for the further protein assay. [1-^14^C] FAs uptake was calculated from the total radioactivity in Cells, ^14^CO2 andASP.

### Lipid extraction and radiolabelled lipid class analysis

Total lipids from cells were extracted according to Folch et al. (1957). The chloroform phase with BHT (0.7 mg/ml) was dried under N_2_ and the residual lipid extract was redissolved in 20 μl chloroform and was applied to the TLC-plate (Merk HPTLC Silica gel 60 F254, 10*20 cm). Phospholipid (PL), free fatty acid (FFA), diacylgycerol (DAG), triglycerol (TAG) and cholesterol ester (CE) were separated by TLC using a mixture of hexane, diethyl ether and acetic acid (85:15:1, v/v/v) as the mobile phase. The different spots corresponding to the lipid classes were scraped off into scintillation vials and the radioactivity was counted in the scintillation counter (LS6500 Beckman Coulter, Brea, CA, USA).

### ATP and triglyceride assay

Cellular ATP levels were assessed by using a Cell Titer-Glo Luminescent Cell Viability Assay kit (Promega, Madison, WI, USA). Triglyceride contents were assayed with EnzyChrom™ Triglyceride Assay Kit (BioAssay Systems, Hayward, CA, USA).

### Western blotting analysis

The solubilized protein from adipocytes was fractionated on 10% SDS-polyacrylamide gels. Gels were transferred to polyvinylidene difluoride (PVDF) membranes. After incubation with 5% nonfat milk for 1h at room temperature, membranes were incubated with primary antibodies overnight at 4°C. Levels of proteins was immunoblotting using the following primary antibodies: Total OXPHOS Rodent WB Cocktail (Abcam, USA), UCP1 (Abcam, USA) and β-actin (Abcam, USA); Secondary antibodies were HRP-conjugated antimouse, antigoat and antirabbit IgG (Santa Cruz, USA). Signals were detected by chemiluminescence (ECL Plus detection system, Clinx science instruments, China) and signals were quantified using Scion Image software (Scion Corporation, USA).

### RNA extraction and quantification of gene transcripts

Total RNA was extracted from the adipocytes using Trizol Reagent (Invitrogen Life Technologies, Carlsbad, CA). One micrograms of total RNA was reverse-transcribed into cDNA using M-MuLV reverse transcriptase kit (Fermentas, EU, Glen Burnie, Maryland, USA). The gene transcripts levels were measured in the ABI Step-One Plus™ Real-Time PCR System (Applied Biosystems, Foster City, CA, USA) according to the procedure described by Wang et al. (1). Data were analyzed by using 2^−ΔΔCt^ and are referred to the W-SAT (SAT from WT mice) using 18S as a reference gene. All primers used in this manuscript were listed in Table 1.

**Table 1:** Specific primers for real-time quantitative PCR

Gene	Primer sequence (5′ to 3′)
PPARγ-F	TGGGTGAAACTCTGGGAGATTC
PPARγ-R	AGAGGTCCACAGAGCTGATTCC
C/EBPα-F	GGTTTCGGGTCGCTGGATCTCTAG
C/EBPα-R	ACGGCCTGACTCCCTCATCTTAGAC
FABP4-F	GACGACAGGAAGGTGAAGAG
FABP4-R	ACATTCCACCACCAGCTTGT
ACBP-F	TTTCGGCATCCGTATCACCT
ACBP-R	TTTGTCAAATTCAGCCTGAGAC
ACSL1-F	CGAGGGCGAGGTGTGT
ACSL1-R	GTGTAACCAGCCGTCTTTGTC
FATP1-F	TCACTGGCGCTGCTTTGGTT
FATP1-R	TCACTGGCGCTGCTTTGGTT
COXIV-F	CGGCGTGACTACCCCTTG
COXIV-R	TGAGGGATGGGGCCATACA
18S-F	AGGGGAGAGCGGGTAAGAGA
18S-R	GGACAGGACTAGGCGGAACA

### Statistics

The significance of the differences between all of the groups was analyzed by one-way ANOVA or t-test. *P* value of <0.05 was considered significant.
